The article "A Clinical Study on the Treatment of Recurrent Chiari (Type I) Malformation with Syringomyelia Based on the Dynamics of Cerebrospinal Fluid" was published in 2022. Journal: Biomed Res Int.

# A Clinical Study on the Treatment of Recurrent Chiari (Type I) Malformation with Syringomyelia Based on the Dynamics of Cerebrospinal Fluid

**DOI:** 10.1155/2022/9770323

**Published:** 2022-10-13

**Authors:** Yongli Lou, Jichao Yang, Haoyuan Gu, Guanghua Xu, Shanfeng Ji, Chi Xu, Yong Liu

**Affiliations:** ^1^Department of Neurospine Surgery, Zhengzhou Central Hospital, Zhengzhou University, Zhengzhou 450000, China; ^2^Xinxiang Medical University, Xinxiang 453003, China; ^3^Yuquan Hospital of Tsinghua University, Beijing 100049, China

## Abstract

**Objective:**

Combining the dynamics of cerebrospinal fluid, our study investigates the clinical effects of syringomyelia after the combination of fourth ventricle-subarachnoid shunt (FVSS) for recurrent Chiari (type I) malformations after cranial fossa decompression (foramen magnum decompression (FMD)).

**Methods:**

From December 2018 to December 2020, 15 patients with recurrent syringomyelia following posterior fossa decompression had FVSS surgery. Before and after the procedure, the clinical and imaging data of these individuals were retrospectively examined.

**Results:**

Following FVSS, none of the 15 patients experienced infection, nerve injury, shunt loss, or obstruction. 13 patients improved dramatically after surgery, while 2 patients improved significantly in the early postoperative period, but the primary symptoms returned 2 months later. The Japanese Orthopedic Association (JOA) score was 12.67 ± 3.95, which was considerably better than preoperatively (*t* = 3.69, *P*0.001). The MRI results revealed that the cavities in 13 patients were reduced by at least 50% compared to the cavities measured preoperatively. The shrinkage rate of syringomyelia was 86.67% (13/15). One patient's cavities nearly vanished following syringomyelia. The size of the cavity in the patient remain unchanged, and the cavity's maximal diameter was significantly smaller than the size measured preoperatively (*P* < 0.001) PC-MRI results indicated that the peak flow rate of cerebrospinal fluid at the central segment of the midbrain aqueduct and the foramen magnum in patients during systole and diastole were significantly reduced after surgery (*P* < 0.05).

**Conclusion:**

After posterior fossa decompression, FVSS can effectively restore the smooth circulation of cerebrospinal fluid and alleviate clinical symptoms in patients with recurrent Chiari (type I) malformation and syringomyelia. It is a highly effective way of treatment.

## 1. Introduction

The clinical signs of syringomyelia (SM) are motor and sensory problems related to the degree of emptiness and spinal cord injury (SCI), with an incidence of around 8.4/100,000. According to relevant pathology, there are five subgroups based on the classification by clinical diagnosis and clinical treatment guidance [1–3]. Approximately 75% of people with SM have Chiari malformation, particularly Chiari I malformation (CM I), the most prevalent type [4]. Since the pathophysiology of SM is unknown, the majority of researches concentrate on cerebrospinal fluid (CSF) dynamics as opposed to anatomical correlations. Consequently, an examination of changes in CSF hydrodynamic parameters in patients with SM is essential for a full assessment of patient circumstances [5–8]. FMD, the first-line therapy approach for SM that improves the stenosis of CSF channels in the subarachnoid cavity, has a favorable postoperative outcome in 80-90 percent of patients [9–13]. However, 14.3% of them reported neurological deterioration within 5 years and 15.4% within 10 years, with the severity of neurological symptoms associated with the grade of arachnoid lesions [14]. As shown in other researches, 30–50% of patients with CM getting FMD may require additional treatment due to persistent, progressive, or recurrent SM [15]. It was suggested to be conservative [16] and not to undergo additional operations for failed imaging reviews but relieved clinical symptoms after FMD, but powerless for the recurrence of SM [17, 18]. According to the literatures [19–21], some specialists recommended shunts for the treatment of these patients, such as syringo-subarachnoidal shunt [22], syringo-peritoneal shunt [23], and syringo-thoracic shunt [24, 25]. Despite the advantages of faster symptom recovery and fewer complications, shunt is rejected for postoperative infection and recurrence of SM caused by shunt blockage [26]. However, it has been reported in the literature that FVSS has the potential to effectively improve the success rate of operation and reduce the risk of excessive CSF drainage as it is able to maintain the integrity of arachnoid and subarachnoid cavity [27]. Despite the above research, FVSS in combination with CSF hydrodynamics is rarely studied in the literature. This paper is the first study to assess CSF dynamics before and after FVSS to investigate the clinical effects of FVSS on recurrent SM by PC-MRI, accumulating clinical experience for the treatment of recurrent SM following FMD.

## 2. Materials and Methods

### 2.1. General Materials

A retrospective analysis studied the clinical data of 15 patients with SM who received FVSS for postoperative recurrent cranial fossa decompression from December 2018 to December 2020. Among 7 men and 8 women, aged between 27 and 59 (mean: 43.8), with a disease duration from 5 to 12 years (mean: 7.1 years). The following are the inclusion criteria: (1) adult patients with SM receiving another infeasible treatment for postoperative recurrent cranial fossa decompression, (2) SM recurrence with neuroprogressive damage, (3) preoperative cerebrospinal fluid examination showing no chronic inflammation or more protein content, and (4) patients and their family members who voluntarily sought FVSS after understanding its aim, risks, and effects.  Table 1 displays preoperative clinical symptoms and their proportion of patients. For the preoperative evaluation made by the Japanese Orthopedic Association (JOA), the 15 patients got a score of 6~13 (mean: 9.86 ± 2.20).

### 2.2. PC-MRI Scan

When scanning, a Siemens Skyra 3.0T superconducting MRI machine was used. Under retrospective ECG gating, the central segment of the mesencephalic aqueduct and foramen magnum was selected for PC-MRI of the head and neck. To set the scan parameters, axial imaging measures the CSF flow rate with a layer thickness of 6 mm, TR 38~50 ms, TE 5.7 ms, one collection, flip angle 30°, matrix 256 × 238, and flow rate encoding (Venc) 22 cm/s. The median sagittal imaging was selected to observe dynamic changes in CSF flow, with a layer thickness of 6 mm, TR 20.36 ms, TE 6.12 ms, one collection, flip angle 10°, matrix 256 × 238, and flow rate encoding (Venc) 22 cm/s. In PC-MRI imaging, high signal indicates downward movement of systolic CSF, signal intensity indicates CSF flow rate (Figure 1(a)), and low signal indicates headward movement of diastolic CS (Figure 1(b)).

### 2.3. Operative Method

All patients were general anesthesia, left lateral decubitus, fixed with a three-nail head frame, fully extended to expose the cervical occipital region. After conventional disinfection and draping, the dissection of atlantooccipital fascia locates the position at 3 cm below occipital bone tuberosity at the hairline in posterior occiput. Under the layer-by-layer longitudinal incision of about 2 cm, posterior edge of foramen magnum as well as congenital absence of posterior arch of atlas was exposed. To decompress the soft tissue, atlantooccipital fascia was detachment, followed by muscle tissue hemostasis. Longitudinal incision of dura mater and arachnoid and bilateral suspension of dura mater were carried out to search the membranous adhesion and obstruction at the export of the 4th ventricle. Upon the incision of adhesive arachnoid, CSF flew out from the 4th ventricle (Figure 2(a)). One end of CSF shunt was placed in the subarachnoid cavity and the other in the 4th ventricle (Figure 2(b)). The suture (PROLENE W8304 7-0) passed through the tough side of the hole tube (SOPHYSA B905S) and then was fixed to arachnoid (Figure 2(c)), and then, it was washed with saline till it became clear. The arachnoid and dura mater were stitched (Figure 2(d)). Color ultrasound exploration was used for accurate positioning (Figure 2(e)). After hemostasis within operational sight, incisions were sutured layer by layer, representing the completion of operation. All procedures were performed by the same skilled surgeon.

### 2.4. Postoperative Evaluation

Postoperative follow-up period ranged from 6 months to 2 years (mean: 11.2 months) during which routine MRI and PC-MRI were performed as a part of reexamination to evaluate the postoperative changes in SM and CSF hydrodynamics. Chicago Chiari Outcome Scale (CCOS) score assesses patients' conditions [28]. The maximum cross-section diameter of syringo was measured before and after FVSS. JOA scores of patients reflect their postoperative neurological improvement.

### 2.5. Statistical Method

Data analysis was performed using SPSS21.0 statistical software based on measurement data expressed as the mean ± standard deviation count data as percentage and *t*-test for comparisons between groups. *P* < 0.05 was considered statistically significant.

## 3. Results

### 3.1. Postoperative Clinical Improvement

No patient had postoperative infection, neurological injury, shunt shedding, or blockage. 13 patients' symptoms were significantly relieved, while 2 patients' early symptoms were greatly relieved as their primary symptoms appeared in the 2^nd^ month after FVSS without further aggravation. CCOS score evaluates the prognosis of patients with SM. Accordingly, patients were divided into the good prognosis and poor prognosis groups with 10 [29] as the cut-off point [29], including 12 with CCOS score > 10 and 3 with CCOS ≤ 10. No symptom deterioration was observed in postoperative patients. The incubation period for onset of symptom improvement varied from 15 days to 3 months. Compared with scores before FVSS, JOA scores of patients after FVSS, ranging from 9 to 16 (mean: 12.67 ± 3.95), were significantly improved (*t* = 3.69, *P* < 0.001).

### 3.2. Postoperative MRI

It was found that MRI of all patients in the 6th month after FVSS had significantly reduced syringo in 13 patients, at least 50% smaller than that before FVSS, a reduction rate of 86.67% (13/15), unchanged syringo in 2 patients, and no syringo progression in any patient. The 2^nd^ MRI of 13 patient in the 24^th^ month after FVSS found a smaller and almost disappeared syringo (Figure 3) in 1 patient than what had been observed in the 6^th^ month after FVSS, with no further changes in the rest of the patients. Statistical results (Table 2) indicated that the maximum diameter of syringo decreased significantly (*P* < 0.001) after shunt.

### 3.3. CSF Flow Rate before and after FVSS by PC-MRI

PC-MRI scans indicated favorable fixing of the shunt in the 4th ventricle-subarachnoid cavity (Figure 4(b)). In the PC-MRI results after FVSS, more intense high-intensity signals in the dorsal and ventral systolic brainstem (Figures 4(c) and 4(d)) were found, suggesting better CSF circulation after FVSS than before FVSS.  Figure 5 shows the systolic peak flow curve of CSF in mesencephalic aqueduct central segment and the systolic peak flow curve of CSF in the foramen magnum, as well as the diastolic peak flow velocity curve of CSF in these two places, respectively. By comparing these four curves, it is found that both systolic and diastolic peak flow velocities significantly decreased (*P* < 0.05) (Table 2 and Figure 5) after FVSS, which was also indicated by quantification results.

## 4. Discussion

There is still a great controversy about shunt for treatment of SM, as there are only small samples evaluated by few studies. Since there is no reliable and consistent criteria, debates continue about which procedure is better for patients, and the clinical history and physical examination of patients still need considering [30]. Different types of shunts have achieved desirable clinical results, at least in the early postoperative period. The current shunt for SM is performed by inserting the shunt into the innermost of syringo to connect to subarachnoid cavity, abdominal cavity, or thoracic cavity, thereby ensuring a better decompression. Peritoneal-shunt offers an option as the absorption capacity is strong due to large negative pressure in low pressure environment. However, the most serious CMI cavity happens in cervicothoracic junction, far away from abdominal cavity, and increases the difficulty of operations as greater omentum in abdominal cavity is highly likely to block the shunt, leading to failures of operations [25, 26]. Most academics prefer to perform shunt at pleural cavity for treatment of SM in recent years due to the negative pressure in pleural cavity and good pressure gradients with the pressure in syringo. However, complications such as shunt blockage, pleural infection, torso numbness, or pain after pleural shunt have been reported in the literatures [24, 31]. Subarachnoid cavity, due to its physiological state, is in theory the most appropriate method of shunt. Soleman et al. [10] reported good therapeutic effects in 21 patients with SM undergoing subarachnoidal shunt, such as relieved clinical symptoms. Davidson et al. [1] studied the therapeutic effect of subarachnoidal shunt in 41 patients with SM, believing that subarachnoidal shunt was ideal because of few complications and good clinical results. Riordan and Scott [27] believed that the blocked outflow of CSF from the fourth ventricle played an important role in the recurrence and progression of SM. The membranous structure of Magendie hole, considered to be caused by postoperative scar adhesion, was seen in some patients during surgery, which was consistent with our observation. Riordan and Scott applied stent tubes to these patients and achieved good results.

Questions have been raised about the pathophysiological mechanism of recurrent cavities. A possible explanation for this might be the individual differences in the first surgical selection and recovery ability. Patients requiring secondary surgery come from all over the country, and their first surgery was also performed by local or national experts. The choice of surgical plan is subject to certain subjectivity and experience, and there is no consensus on the need for combined extended duraplasty. Previously, CMI was considered to be a syndrome characterized by posterior fossa stenosis malformation, inferior cerebellar tonsillar hernia resulting in abnormal CSF circulation and subsequent nerve damage, and often accompanied by the occurrence of syringomyelia [32]. FMD improves CSF circulation by increasing the narrow subarachnoid cavity at foramen magnum to ultimately shrink or delay SM progression [12, 33–37]. Expanded duraplasty is commonly used as a supplement to FMD surgery. On the basis of bone decompression, the dura mater is expanded and reconstructed to achieve better decompression effect and restore CSF circulation to a greater extent. Although FMD combined with extended duraplasty [32], arachnoid adhesion lysis and dural reconstruction are all procedures aimed at reconstructing the smooth physiological CSF flow, which improves the clinical remission rate of SM, but increases the risk of complications and recurrence [8, 25, 38, 39]. This may explain why many surgeons only perform FMD. In recent years, structural instability of the craniocervical junction has been proposed as the pathogenesis of CMI, including atlantoaxial instability and atlantooccipital instability. After analyzing 388 clinical cases, Goel et al. [40] proposed to redefine Chiari malformation as Chiari Formation, arguing that syringomyelia was a secondary neurological damage caused by “atlantoaxial instability,” and the decline of cerebellar tonsils was the compensation of the spinal cord itself occurred naturally and stabilized the bony structure of the craniocervical junction as the primary goal of surgery. However, this theory does not address the question of asymptomatic cases or significant morphological evidence of changes in PCF (posterior fossa). Wan et al. [41] believed that atlantooccipital instability caused the decline of cerebellar tonsils and contributed to nerve damage. However, the study did not explain the physiological link. Some studies have proposed concepts such as craniocervical junction compliance to try to explain the phenomenon, but yet no mechanism or theory has been found to be the perfect explanation.

In general, FVSS ensures the relative patency of cerebrospinal fluid circulation, benefiting patients with secondary surgery as our surgical results show, which further confirmed the opinion of Goel et al. [40] and Riordan and Scott [27] that FMD is indeed good for Chiari patients. SM may be related to complications such as cerebellar tonsillar ptosis, tissue adhesion, and atlantoaxial instability, so secondary surgery will be effective. As a result, the circulation of cerebrospinal fluid in the craniocervical junction is of great significance to the occurrence of the disease. FVSS surgery has been proposed in recent years as a salvage measure for postoperative recurrence of FMD, but related clinical studies are few. In addition to shunt surgery, atlantoaxial fixation is also a surgical option [40]; however, it appears that extended duroplasty cannot be performed alone or as the best salvage measure [32]. Naturally, apart from patients with atlantoaxial fixation, the motion range of neck is greater. For patients at the age of 27-59 years (average age: 43.8 years), the “stability” of the dural structure will face greater challenges, especially in patients with secondary surgery. Recurrence is surely regrettable. The physical properties of the shunt pipe material, such as hardness, flexibility, and ability to resist the oppression, are stronger than those of the epidural. Although the PC-MRI waveform in the study (Figure 5) showed that the surgery did not completely restore the CSF circulation of the patient, it could provide the patient with a relatively stable CSF circulation. From the perspective of recurrence risk, we believe that FVSS may be a better choice, and it is also a bold choice for the current surgical treatment of Chiari deformity.

However, our study found that FVSS can improve CSF circulation in subarachnoid cavity at foramen magnum without damaging the spinal cord. It is applicable to patients with idiopathic SM and patients with great risks of operation by secondary needling manipulation following ineffective treatment of protopathy. Despite the apparent effects of syringo-subarachnoidal shunt reported by Davidson et al. [1] in such patients, we believe that patients may be at risk of postoperative spinal cord-related nerve injury, shunt shedding, or blockage. FVSS can be used as a complementary treatment for recurrent SM. For 15 patients with recurrent SM or aggravated symptoms after FMD, we chose FVSS with small risks and few complications owing to great risks of possible neurological damage and vascular damage after local adhesion lysis [14]. No patient experienced postoperative infection, neurological injury, shunt shedding, or blockage. We ruled out the risk of shunt blockage caused by increased CSF protein through the preoperative assessment of the cerebrospinal fluid properties. Meanwhile, the surgery followed strict aseptic operation to avoid the blockage of the shunt tube that might be caused by inflammation and strictly controlled the hemostasis with the aid of a microscope, so as to reduce the blood entering the cerebrospinal fluid as much as possible. After the operation, antibiotics should be given prophylactically, and the surgical wound should be taken cared closely to prevent complications such as CSF leakage and infection. According to the hydrodynamic characteristics of cerebrospinal fluid, the shunt was placed in the fourth ventricle and subarachnoid space, preventing nerve damage. When the shunt tube is fixed, the mobility (0.5 cm) is indwelled appropriately according to the preoperative PC-MRI cerebrospinal fluid dynamic parameters and intraoperative ultrasound, thus preventing the shunt tube from falling off to a certain extent. To date, no blockage or displacement of the shunt tube has been found in the postoperative follow-up of the patient, and we will follow up the condition regularly.

The schematic diagram of the fixing method of the shunt pipe is shown in Figure 6.

After shunt, 13 patients showed greatly relieved symptoms, and early symptoms were significantly relieved in 2 patients whose primary symptoms appeared in the 2nd month after FVSS without further aggravation. The MRI for all patients in the 6th month after FVSS indicated that syringo has been significantly reduced in 13 patients by at least 50% compared to that before FVSS, representing a reduction rate of 86.67% (13/15). However, 2 patients have unchanged syringo and no syringo progression in any patient. The second MRI of 13 patients in the 24th month after FVSS found a smaller and almost disappearing syringo (Figure 3) in 1 patient compared to the MRI results in the 6th month after FVSS. There are no further changes in the rest of the patients. Statistical results (Table 2) indicated that the maximum diameter of syringo decreased significantly (*P* < 0.001) after shunt, indicating that FVSS had a significant effect on recurrent CMI after FMD.

PC-MRI is known for its noninvasiveness, multiplane imaging, and high sensitivity to slow fluid. It is widely used in CSF hydrodynamics evaluation after NPH, CMI, SM, and neurosurgery, so the technique is gradually used in the qualitative and quantitative study of CSF hydrodynamics [42, 43]. Previous related studies described SM as a pathological sign of disordered CSF dynamics caused by anatomical abnormalities at craniocervical junction. Tosi et al. [16] and Riordan and Scott [27] suggested that SM recurrence after FMD is associated with abnormal CSF circulation, although there has been little agreement on the pathophysiological mechanisms of asymptomatic cavity patients and patients with successful but poor radiological outcomes after cavity surgery. The description of low velocity fluids in a complex physiological environment within the craniocervical junction has been troubling to clinical researchers. Unlike Gholampour and Fatouraee [44] and Frič and Eide [45], who aimed to build a complete central nervous system model to simulate real CSF dynamics, more researchers focus on the description of local CSF flow. In the studies of the driving forces of CSF dynamics, Xu et al. [46, 47] suggested that head movement is one of the important driving forces of CSF circulation. However, Daouk et al. [48] and Dreha-Kulaczewski et al. [49] studied the effect of respiratory movement on the spatial propagation characteristics of intracranial CSF, believing that respiratory movement is the most important driving force of human CSF flow. Daouk et al. [48] noted that cardiac beating has a larger influence on CSF flow rate than respiratory movement, but respiratory movement makes CSF shift farther. In the studies of CSF abnormalities at the craniocervical junction, Alperin et al. [50, 51] found that the spinal canal affected the spatial distribution of CSF by modulating ICP during body posture changes, and pointed out that the low-pressure craniospinal CSF system was more easily affected by body posture changes than the high-pressure cerebrovascular system. The maximum spinal cord displacement and intracranial volume changes during the cardiac cycle and measures reflecting the cerebral venous drainage pathway may be predictors of decompression outcomes in CMI patients. Tarumi et al. [52] applied PC-MRI to assess changes in CBF and CSF flow dynamics during moderate-intensity rhythmic handgrip exercise in healthy young men and women, suggesting the measured stroke volume of arterial, venous, and venous sinuses is positively correlated with changes in the stroke volume of CSF in the cerebral aqueduct during exercise. In the studies of CSF metabolomics, Fultz et al. [53] found a consistent mode of oscillatory electrophysiology, hemodynamic, and cerebrospinal fluid dynamics in NREM sleep from the perspective of physiological and neural dynamics of the brain. They also proposed how neurodynamics and hemodynamic rhythm correlate with CS fluid dynamics. As they suggested, the sleeping brain shows CSF flow waves on the macroscale, providing a new perspective for CSF dynamics research. In recent years, Labuda et al. [54] proposed the concept of “craniocervical junction compliance,” which connects the driving force of CSF with abnormalities in local central nervous system, further explaining syringo-related clinical phenomena. Despite the great development of noninvasive imaging techniques from iodooil radiography to PC-MRI, an accurate and complete description of low velocity fluids in a complex physiological environment is still difficult to obtain and insufficient to fully explain current clinical phenomena. Therefore, we focused on changes of CSF dynamics in subarachnoid cavity before and after FVSS, hoping to provide additional support to today's clinical studies.

Abnormalities of CSF dynamics in subarachnoid cavity in CMI patients are more pronounced in the presence of SM. Studies have reported [55] that the flow rate (ml/min) of CSF flowing through the foramen magnum depends on cerebral blood volume during each cardiac cycle, and it is largely decided by the size and shape of foramen magnum. Any process limiting flow within the foramen magnum may increase CSF flow rate. In this study, PC-MRI measurements showed that CSF flow was bidirectional in the central segment of mesencephalic aqueduct and foramen magnum. The systolic and diastolic peak flow velocities were significantly lower than those before FVSS, indicating a dramatic improvement in CSF flow rate. Gholampour and Taher [7] studied the CSF hydrodynamics in 41 patients with SM and 18 healthy people, finding that the curve of CSF flow rate of all patients in the cardiac cycle is a regular and smooth sine wave-like curve, similar to the conclusion of Rutkowska et al. [56] and Takizawa et al. [57]. In contrast, the curve of CSF flow rate after FVSS is chaotic, which is inferred to be due to the impact of shunt implantation. At subsequent follow-ups, we grouped patients with different prognostic outcomes according to CCOS score and found that symptoms were significantly relieved. The syringo became smaller in 13 patients with higher CCOS score while 2 patients with lower CCOS scores have the same primary clinical symptoms and slightly changed syringo. In PC-MRI, CSF peak flow rate in central segment of mesencephalic aqueduct and foramen magnum also improved significantly, consistent with CCOS score, further proving the strong correlation between improvement in CSF dynamics and clinical outcome. Hence, FVSS can evaluate patient prognosis in synergy with CCOS score. Therefore, we inferred that patients after FVSS can effectively restore the smooth CSF circulation, achieving a good clinical effect.

## 5. Conclusion and Limitations

For patients with persistent and recurrent SM after FMD, FVSS is a safe and effective operative treatment program in the event of poor treatment effects that cannot be addressed clinically. In addition, FVSS can effectively evaluate operative and prognostic effects in combination with CSF dynamics.

There are many limitations to our study, such as retrospective analysis and small cohort of patients. Furthermore, the time of clinical follow-up varied greatly in our study, which may be one of the reasons for the biased results. The long-term effect of FVSS still needs to be evaluated through longer-term follow-ups. We hope to have the opportunity to cooperate with multiple regional medical centers to carry out large-scale prospective studies in the future. We wish that FVSS could bring new hope to patients with recurrent Chiari (type I) deformity combined with syringomyelia.

## Figures and Tables

**Figure 1:** PC-MRI images ((a) high signal indicates downward movement of systolic CSF (as indicated by the red arrow); (b) low signal indicates headward movement of diastolic CSF (as indicated by the red arrow)).

**Figure 2:** FVSS intraoperative pictures.

**Figure 3:** Preoperative and postoperative imaging data of CMI patients ((a–c) preoperative MRI; CMI patients after FMD (arrow in (b)), sagittal position, and cross section indicate large syringo in cervicothoracic junction; (d–f) MRI in the 6th month after FVSS (arrow in (d) indicates shunt position) found a significantly reduced syringo; (g–i) the 2nd MRI of patients in the 24th month after FVSS found a smaller and almost disappeared syringo than that observed in the 6th month after FVSS. (c, f, and i) represent the maximum cross-section of syringo).

**Figure 4:** PC-MRI scans.

**Figure 5:** Curves of systolic peak flow of CSF in central segment of mesencephalic aqueduct before and after FVSS and curves of diastolic peak flow velocities of CSF in foramen magnum before and after FVSS.

**Figure 6:** Diagram of shunt tube fixation.

**Table 1:** Preoperative clinical symptoms of 15 patients.

Symptom	Number of people (person)	Proportion (%)
Cervicodynia	12	0.80
Myophagism	9	0.60
Convulsion	8	0.53
Numbness of limbs	10	0.67
Decreased upper extremity strength	8	0.53
Decreased lower extremity strength	8	0.53
Nystagmus	5	0.33
Dissociative sensory disturbance	7	0.47
Gait disorder	3	0.20
Dysphagia	2	0.13

**Table 2:** Comparison of relevant parameters before and after FVSS ($\bar{x}\pm s$).

	Maximum diameter of syringo (mm)	JOA	Foramen magnum		Central segment of mesencephalic aqueduct	
			Systolic peak flow velocity (cm/s)	Diastolic peak flow velocity (cm/s)	Systolic peak flow velocity (cm/s)	Diastolic peak flow velocity (cm/s)
Before FVSS	10.50 ± 2.55	9.86 ± 2.20	7.06 ± 1.56	7.18 ± 2.86	6.82 ± 2.25	6.22 ± 2.15
After FVSS	5.08 ± 2.43	12.67 ± 3.95	5.50 ± 1.22	5.92 ± 1.62	5.41 ± 1.86	5.24 ± 1.12
*t*	5.29	3.69	4.03	4.33	5.73	6.32
*P*	*P* < 0.001	*P* < 0.001	*P* < 0.01	*P* < 0.05	*P* < 0.05	*P* < 0.05

## Data Availability

The datasets used and/or analyzed during the current study are available from the corresponding author on reasonable request.
